# Treatment of melasma in Caucasian patients using a novel 694-nm Q-switched ruby fractional laser

**DOI:** 10.1186/2047-783X-18-43

**Published:** 2013-11-14

**Authors:** Said Hilton, Heike Heise, Bettina Alexandra Buhren, Holger Schrumpf, Edwin Bölke, Peter Arne Gerber

**Affiliations:** 1 Medical Skin Center, Düsseldorf, Germany; 2 Departments of Dermatology, University of Düsseldorf, Düsseldorf, Germany; 3 Radiation Oncology, Medical Faculty, University of Düsseldorf, Düsseldorf, Germany

## Abstract

**Background:**

Melasma is a common hypermelanosis of the face. The use of a classical Q-switched ruby laser (QSRL) to treat melasma is discussed controversially and is associated with frequent adverse effects, such as hyper- or hypopigmentation. Recently a fractional-mode (FRx) QSRL was developed to minimize the adverse effects of classical QSRL. The objective of this research was to evaluate the efficacy and safety of a novel FRx-QSRL in the treatment of melasma in Caucasian patients.

**Methods:**

We performed a retrospective study of 25 Caucasian melasma patients (Fitzpatrick skin types I to III). Patients received one to three FRx-QSRL treatments (Tattoostar FRx, Asclepion Laser Technologies, Jena, Germany) at pulse energies of 4 to 8 J/cm^2^. Three blinded investigators independently evaluated the melasma area and severity index (MASI) score before treatment and at the four- to six-week follow-ups. At additional three-month follow-ups, patients evaluated subjective improvement, pain and over-all satisfaction with the treatment according to a numeric analogue score (NAS). Side effects were documented.

**Results:**

At four to six weeks post laser treatment for a mean of 1.4 sessions, we observed a significant (*P* = 0.0001) reduction of the MASI score from 6.54 to 1.98 (72.3%). Patients rated the pain of the intervention at a mean 2.46 points (0 = no pain; 10 = maximum pain), the improvement at a mean 5.55 points (0 = no improvement; 10 = maximum improvement) and the overall satisfaction at a mean 4.66 points (0 = not satisfied; 10 = maximum satisfaction). After three months, post-inflammatory hyperpigmentation (PIH) and/or recurring melasma were observed in 7 (28%) and 11 (44%) patients, respectively.

**Conclusion:**

The 694-nm FRx-QSRL is a safe and effective option for treating melasma in Caucasian patients. Over periods of >3 months, PIH and/or recurring melasma may develop at significant rates and may reduce patient satisfaction. Multiple treatment sessions with lower pulse energies and/or a post-interventional therapy with hypopigmenting ointments and UV protection may help to minimize these complications.

## Background

Melasma is a common acquired benign pigmentary disorder that classically manifests as symmetrical hypermelanosis of the face. Most commonly melasma affects women of reproductive age with darker skin types (Fitzpatrick skin types IV and higher) but it may also occur at other ages and in men. Briefly, the Fitzpatrick skin type classification system is based on the color of the skin (type I being the fairest (white) and type VI being the darkest (black)) and its response to UV exposure (pigmentation) [1]. An estimated more than five million people are affected by melasma in the United States of America alone [2]. Melasma has a significant negative impact on a patient’s quality of life [3]. Risk factors include ultraviolet (UV) exposure, hormonal alterations (for example, pregnancy or oral contraceptives), thyroid disease and anti-seizure medication. Melasma that is related to pregnancy (or hormonal alterations) is also referred to as chloasma.

The pathogenesis of melasma has remained largely elusive. Established concepts propose a stimulation of pigment-producing cells (melanocytes) by sex hormones (estrogen and progesterone) and UV irradiation. Recent studies have reported paracrine effects amongst melanocytes, keratinocytes and/or fibroblasts [4-7], and have identified stem cell factor (SCF) and c-kit as pathogenic factors. The authors propose that UV irradiation induces SCF in dermal fibroblasts. Subsequently, the proliferation and melanogenesis of melanocytes is induced via SCF/c-kit-induced signaling [8]. Hypopigmenting topical agents containing hydroquinone, broad-spectrum UV protection and camouflage are considered the current standard of care for treating melasma. Additional therapeutic options include topical retinoic acids (tretinoin), azelaic acid, microdermabrasion, chemical peeling or electromagnetic devices, such as lasers [9-12].

Various laser and light systems, including ruby lasers, Er:YAG lasers, carbon dioxide (CO_2_) lasers and intense pulsed light (IPL), have been evaluated for their efficacy in treating melasma [12-14]. IPL therapy effectively reduced the severity of melasma in a population of 89 Asian women [15]. The use of conventional ablative laser systems (Er:YAG and CO_2_) for treating melasma has been reported to be associated with a significant frequency of post-interventional hyper- as well as hypopigmentation [16,17]. The frequency of adverse effects may be limited by using novel fractional laser systems [18]. Notably, several trials studying the effects of Q-switched ruby lasers (QSRLs) have reported controversial results. In 1994, Taylor and Anderson noted that QSRLs were ineffective for treating refractory melasma and post-inflammatory hyperpigmentation [19]. A split-face study by Tse *et al*. demonstrated that melasma patients developed post-inflammatory hyperpigmentation (PIH) and worsening of the melasma after QSRL therapy [20]. Conversely, a recent study by Jang *et al*. reported that a novel fractional-mode (FRx) QSRL (Tattoostar FRx, Asclepion Laser Technologies, Jena, Germany) may be effective in treating melasma in Korean patients [21].

Fractional photothermolysis has revolutionized laser resurfacing (LSR) and was initially presented by Manstein and coworkers in 2004 [22]. The significant adverse effects of classical LSR are significantly reduced by delivering the laser beam using a microarray. This technique creates microscopic columns of treated tissue and intervening areas of untreated skin, thereby allowing rapid re-epithelialization and minimal downtime. Fractional delivery has been developed for CO_2_, Er:YAG, and yttrium scandium gallium garnet lasers [23]. Recently, a fractional-mode QSRL has been developed (Tattoostar FRx, Asclepion Laser Technologies, Jena, Germany), which can homogeneously deliver ruby laser microspots. The laser delivers a 7.1 × 7.1 mm^2^ array of 196 microspots of 300 μm at a pulse duration of 40 ns, with an overall coverage of 27.7%. This approach may minimize the adverse effects of classical QSRL, such as PIH and hypopigmentation. Here, we present a retrospective analysis of 25 Caucasian patients, which assesses the efficacy of an FRx-QSRL in treating melasma.

## Methods

### Patients

In the study, 25 Caucasian women (mean age 39.8 years; range 31 to 57; Fitzpatrick skin types I to III) with melasma were treated with an FRx-QSRL (Tattoostar FRx, Asclepion Laser Technologies, Jena, Germany) at the Medical Skin Center, Düsseldorf, in 2010 and 2011. Patients presented with epidermal or mixed-type melasma. Of the patients, 19 had had melasma <10 years and 6 had had it >10 years. The melasma areas were located on the forehead (*n* = 14), the cheeks (*n* = 12), the chin (*n* = 2) or the upper lip (*n* = 2). Identified risk factors included past pregnancies (*n* = 5), hormonal therapy (*n* = 12) and UV exposure (*n* = 25). Some patients presented with melasma in multiple locations and/or risk factors.

### Treatment

We used a 694-nm FRx-QSRL (Tattoostar FRx, Asclepion Laser Technologies, Jena, Germany) at fluences of 4 to 8 J/cm^2^ and a frequency of 1 Hz. For each individual patient, the fluence was gradually increased to identify the minimal fluence needed to achieve a clinical effect (photosdisruption). Each patient received laser treatment for all affected areas. In pain-sensitive patients, a topical anesthetic (a lidocaine-tetracaine mix) was applied onto the treated areas 30 minutes prior to treatment. However, most patients tolerated the intervention without anesthesia. The laser treatment lasted up to 10 minutes depending on the size and number of treated areas. Post-intervention, cool packs were applied. Patients were advised to use strict UV protection. If more than one treatment was needed, the patient received additional treatments after intervals of four weeks.

### Evaluation

Photographs (Canon EOS 40D digital camera, Tokyo Japan) were taken before therapy and at the four- to six-week follow-up sessions. Three blinded investigators independently evaluated the melasma area and severity index (MASI) score before treatment and at the four- to six-week follow-ups, as previously described [24]. At the additional three-month follow-ups, patients evaluated subjective improvement, pain and their overall satisfaction with the treatment was determined according to a numeric analogue score (NAS). At this time point, side effects were documented.

### Statistical analysis

Student’s T-test was used for the statistical analysis, and *P* < 0.05 was regarded as statistically significant.

## Results

The analysis included 25 patients. At the follow-up at four to six weeks after the last treatment (there were up to three treatment sessions with a mean of 1.4 sessions) the average MASI score showed a significant reduction from 6.54 to 1.98 (72.3%) (Figures 1 and 2). In general, the adverse effects for the first days post therapy were mild and included erythema, a burning sensation, pruritus and exfoliation. After three months, PIH and/or recurring melasma were observed in 7 (28%) and 11 (44%) patients, respectively.

**Figure 1:** **Melasma in Caucasian patients before and four to six weeks after one treatment with the 694-nm FRx-QSRL. (a)** 39-year old woman, fluence 6 J/cm^2^, front: 2 passes, cheeks: 1 pass. **(b)** 42-year-old woman, fluence 6 J/cm^2^, 1 pass. **(c)** 51-year-old woman, fluence 6 J/cm^2^, 2 passes. **(d)** 42-year-old woman, fluence 5 J/cm^2^, 1 pass. Presented cases are representative examples of the 25 treated patients. FRx, fractional-mode; QSRL, Q-switched ruby laser.

**Figure 2:** **Melasma area and severity index (MASI) scores before and four to six weeks after the final treatment with the 694-nm FRx-QSRL.** Values are plotted as individual ratios and mean ratios are shown by the horizontal bar (*** *P* ≤ 0.0005). FRx, fractional-mode; QSRL, Q-switched ruby laser.

The patients’ self-evaluation rated the pain of the intervention at a mean 2.46 points (0 = no pain; 10 = maximum pain), the improvement at a mean 5.55 points (0 = no improvement; 10 = maximum improvement) and the overall satisfaction at a mean 4.66 points (0 = not satisfied; 10 = maximum satisfaction). We also used the same protocol to treat patients with darker skin types and melasma and/or PIH, with satisfactory results (Figure 3).

**Figure 3:** **Melasma in an African patient before and 12 weeks after the final treatment with the 694-nm FRx-QSRL.** 50-year old woman; first session: fluence 6 J/cm^2^, 1 pass; second session: fluence 7 J/cm^2^, 1 pass. The patient applied a combination of topical bleaching agents and strict UV protection for the documented 12 post-intervention weeks. FRx, fractional-mode; QSRL, Q-switched ruby laser.

## Discussion

Laser therapy is based on the biophysical principle of selective photothermolysis. The lasers used emit light at a wavelength that is specifically and adequately absorbed by the target chromophores [25]. The target chromophore for pigmented lesions is melanin. Laser light that is adequately absorbed by melanin includes that from ruby (694 nm), Nd:YAG (523 and 1064 nm) and alexandrite (755 nm) lasers. Q-switched (QS) lasers generate a rapid burst of light, which matches the thermal relaxation time for melanin, thereby effectively destroying the pigment [14].

QS-Nd:YAG lasers have been shown to be effective and are widely used in the management of melasma [26-29]. A representative recent study by Zhou *et al*. of 50 patients (Fitzpatrick skin types IV to VI) demonstrated a mean decrease in the MASI score of 61.3% after nine sessions. At the three-month follow-up a recurrence rate of 64% was noted [29]. A study of 50 patients by Sim *et al*. reported improvement rates of 50% to 74% [28]. For the QSRL, earlier reports state that the laser is ineffective for melasma or may even worsen the pigmentation after therapy [19,20]. Conversely, a recent study by Jang *et al*. demonstrated a mean decrease of the MASI score of 29.8% in 15 Korean patients after six treatments with an FRx-QSRL (Tattoostar FRx, Asclepion Laser Technologies, Jena, Germany). Two patients reported a slight worsening. None of the patients reported any long-term adverse effects such as PIH [21]. Jang *et al*. found that a QSRL was more effective for treating melasma compared to a QS-Nd:YAG laser [21]. This has been demonstrated by comparative studies for other pigmented lesions, such as nevus of Ota, lentigo, PIH and Becker’s nevus, and it is proposed that this is due to the stronger absorption of the 694-nm wavelength light (QSRL) by melanin compared to 1064-nm wavelength light (QS-Nd:YAG) [20,21,30].

Consistent with the results of Jang *et al*., we have demonstrated a significant (*P* = 0.0001) decrease of the MASI score of 72.3% in 25 Caucasian patients after a mean of 1.4 sessions with an FRx-QSRL (Tattoostar FRx, Asclepion Laser Technologies, Jena, Germany). As the risk of common adverse effects of QSRL therapy, such as PIH, is expected to be significantly lower in Caucasian compared to Asian skin types, we applied higher fluences (4 to 8 J/cm^2^) per session compared to Jang *et al*. (2 to 3 J/cm^2^). However, this more aggressive treatment resulted in a significantly higher rate of adverse effects (PIH and/or recurring melasma in 28% and 44% of the patients). Lower fluences and multiple treatment sessions may reduce the frequency of these adverse effects. However, many patients refuse further treatment (and want to avoid additional costs) if the result of an initial treatment is minimal. An additional option could be a multimodal therapy using an FRx-QSRL in combination with microdermabrasion [27], chemical peeling [31] and/or hypopigmenting topical agents [32].

## Conclusions

In summary, the FRx-QSRL is a safe and effective treatment for melasma for patients with Caucasian or Asian skin types. Multimodal concepts may further increase the efficacy and reduce the adverse effects of the therapy. We maintained only a three-month follow-up after the final treatment, so further long-term studies are needed.

## Consent

Written informed consent was obtained from the patients for the publication of this report and any accompanying images.

## Abbreviations

FRx: Fractional-mode; IPL: Intense pulsed light; LSR: Laser resurfacing; MASI: Melasma area and severity index; PIH: Post-inflammatory hyperpigmentation; QS: Q-switched; QSRL: Q-switched ruby laser; SCF: Stem cell factor.

## Competing interests

PA Gerber received honoraria for oral presentations by Asclepion Laser Technologies.

## Authors’ contributions

SH and HH performed the laser treatments and collected the data. BAB, HS, EB and PAG evaluated and analyzed the data, and wrote the manuscript. All authors read and approved the final manuscript.
